The article "Evaluating the Performance of Inclusive Growth Based on the BP Neural Network and Machine Learning Approach" was published in 2022. Journal: Comput Intell Neurosci.

# Evaluating the Performance of Inclusive Growth Based on the BP Neural Network and Machine Learning Approach

**DOI:** 10.1155/2022/9491748

**Published:** 2022-06-30

**Authors:** Shuangshuang Fan, Xiaoxue Liu

**Affiliations:** ^1^School of Management, China University of Mining and Technology-Beijing, Beijing 100086, China; ^2^School of Economics, Beijing Technology and Business University, Beijing 100048, China

## Abstract

In this paper, we use the panel data of 281 cities in China from 2005 to 2020 for capturing the factors driving urban inclusive growth (IG). In doing this, we employ the BP neural network algorithm combined with the DEA model to measure the urban inclusive growth efficiency (IGE). Furthermore, a nest of machine learning (ML) algorithms are introduced to explore the drivers of urban IGE, which overcomes the defects of endogeneity and multicollinearity of traditional econometric methods. We find for the overall sample that entrepreneurship and innovation contribute the most to IGE, accounting for about 35%, respectively, and they are the most critical drivers, while the heterogeneity test results reveal that the contribution of influencing factors has changed for different regions such as the eastern region, the central region, and the western region. Based on the experimental results of the ML model, we provide some policy suggestions for China and similar developing countries and emerging economies to promote IG.

## 1. Introduction

In the recent two decades, since the outbreak of the 1998 global financial crisis, inequality has been rising in importance on the global agenda. Inequality of wealth, income, and opportunity, whether within or between countries, has become the focus of attention [1]. The global Gini coefficient has hovered around 0.7 since 1980 and decreased slightly since 2002, while this is a conservative estimate [2]. It will slow down if the income growth rate of the poorest percentile increases faster than that of the richer percentile, even though the absolute gap has widened [3]. According to the report of the World Institute for development economics of the United Nations University, the average income of the richest 1% has increased by 10.1 times in absolute terms compared with that of others since 1980 [4]. To address this situation, the Asian Development Bank (ADB) established a new principle-inclusive growth (IG), which posited that apart from guaranteeing a wide participation and role to the growth procedure, issues of gender, ethnicity, and race and even environment should be part of IG [5–7]. The World Bank on the other hand stated that the issues of fairness of opportunity, social protection, and productive employment as contrasting to short-term income redistribution should be enshrined in IG [7]. This emphasizes economic growth while paying attention to social equity, taking into account benefits and equity, which can be conducive to the realization of the goal of sustainable growth [8]. Thus, a better understanding of IG determinants to develop effective policy responses [9] is in order.

The article "Evaluating the Performance of Inclusive Growth Based on the BP Neural Network and Machine Learning Approach" was published in 2022. Journal: Comput Intell Neurosci.

However, the literature on IG is still relatively limited [6], especially for emerging and developing economies. This paper holds that IG is a development model in which the economic system and the social system are coordinated and efficiency and equity are taken into account. It emphasizes that in the process of economic growth, we should provide general social members with opportunities to receive education and participate in the process of economic growth, such as employment and entrepreneurship, so as to increase their income and narrow the income gap between people. In addition, it also considers that the benefits brought by economic growth are fairly distributed by the society, so as to ensure that social members enjoy social well-being equally. A few studies explain how IG is measured. Some scholars use the income-based measurement method [10, 11], others use the non-income-based measurement method [12, 13], resulting in policy prescriptions based on these theoretical and empirical results that are often controversial. Further, in studying the key drivers of IG, scholars mostly use traditional econometric models and draw different conclusions. For instance, Whajah et al. [14] used a fixed effect regression model to examine the relationship between government size, public debt, and IG for a panel of 54 African countries, and found that the former has a positive effect on IG, while the later has a negative effect on IG; Ajide et al. [15] investigated the dynamic relationship between economic globalization, entrepreneurship, and IG using panel econometrics; Biswas et al. [10] proposed foreign direct investment and trade liberalization fostering greater inclusiveness, while financial deepening and technological change have no discernible effect; Kouton [16] examined the role of trade facilitation measures in lowering barriers to trade and raising incomes and promoting IG. Furthermore, Kang and Martinez-Vazquez [17] examined the conditions under which the FDI can effectively lead to IG using a fixed effects regression; Oyinlola et al. [18] explored the relationship between human capital, innovation, and IG by the fixed effects model; Seven [19] employed a series of econometric models to study the relation between financial development and income inequality. Additionally, based on nationwide observations, Wang et al. [20] employed the structural equation model in testing the impact of public housing supply on urban IG in China. These studies explain the determinants of IG from different perspectives and contribute to relevant research, but there are also some potential deficiencies and limitations.

The article "Evaluating the Performance of Inclusive Growth Based on the BP Neural Network and Machine Learning Approach" was published in 2022. Journal: Comput Intell Neurosci.

The first concern of previous research is that the analysis of multivariables is usually based on a large number of highly correlated variables, which may lead to the problem of multicollinearity. More critically, using a broad set of correlated variables in regression models not only yields inconsistent and inefficient coefficient estimates but also poses challenges in the interpretation of these regression-based estimates, and standard econometric methods cannot deal with such a large set of proxy variables. One must typically engage in two steps by first preselecting a small number of variables and then investigating their relationships with the integration metric [21]. In addition, previous studies only focused on the causal relationship between some drivers and IG, while ignoring the predictive ability of the explanatory variables to IG. There are great differences between explanatory models and predictive models in terms of concept and optimization objectives [22, 23]. The influencing factors that have an explanatory power on IG may not accurately predict the IG level. Therefore, it is impossible to draw the conclusion of prediction effect from the estimation results of the causal inference model. To solve these problems, this study introduces a series of Machine Learning (ML) methods, including the Random forest (RF) algorithm, the XGBoost algorithm, the CatBoost algorithm, and the LightGBM algorithm to study the drivers of IG of 281 prefecture-level cities in China. Furthermore, the importance and weight of different drivers will be analyzed. By comparing the results of various ML models, the most suitable for evaluating the driving factors of IG is established and compared with the results of traditional econometric regress models to verify the superior performance of ML to study the drivers of IG for the samples.

Our study makes an important contribution to the existing literature on IG. It uses the BP neural network algorithm and data envelopment analysis (DEA) to measure the level of inclusive growth efficiency (IGE) in 281 Chinese cities from 2005 to 2020. It also reveals multiple factors driving IG. The advantage of the BP neural network is to increase the prediction ability of the evaluation index of IG constructed in this paper. Based on this evaluation model, we can predict the level of urban IG according to the value of the explanatory variables of the city. Contrast to previous literature, which focuses on the influence of a single factor, this paper not only integrates the role of various factors, but also calculates the contribution of various factors in influencing IG. We find that for overall cities, the most critical drivers of urban IGE are entrepreneurship and innovation, accounting for about 35%, respectively, while GDP and innovation are the main driving forces of IG in eastern China, and innovation and FDI are the main driving forces of IG in central and western China. Based on this, the relevant policies to drive IG can grasp the main contradiction and be more targeted. We choose Chinese cities as the research object because the issue of IG is more urgent in China. According to the results of China's household follow-up survey (CHFS), China's Gini coefficient has been higher than the international warning line by 0.4 since 2000, and shows an upward trend year by year. By 2018, it reached 0.468, exceeding the average level of developed countries and emerging economies. If the rising trend of inequality is not restrained, it will cause serious economic and social losses. If the reform were to be blocked and stopped, the growth rate will decline and inequality will become more serious. The absolute gap of social income will lead to social and political tensions and social conflicts. Therefore, we choose to study the driving factors of IG in Chinese cities and put forward targeted policy suggestions, which could provide a reference for China and similar emerging economies and developing countries.

The article "Evaluating the Performance of Inclusive Growth Based on the BP Neural Network and Machine Learning Approach" was published in 2022. Journal: Comput Intell Neurosci.

Additionally, our work also expands the literature on the application of advanced ML techniques in empirical research in economics. For example, Adetunji et al. [24] explored the use of the Random Forest ML technique for house price prediction. Mustafa et al. [25] trained an artificial neural network (ANN) model to recognize the pattern of the financial market and used this model to detect whether and when the market pattern has changed. Ben Jabeur et al. [26] employed a nest of ML, such as the LightGBM, CatBoost, XGBoost, Random Forest (RF), and neural network models, to predict oil prices during the COVID-19 pandemic. Richardson et al. [27] evaluated the real-time performance of popular ML algorithms in obtaining accurate nowcasts of real GDP growth for New Zealand. We advance this line of research by applying the ML technique to circumvent the multicollinearity issue in determining the drivers of the urban IG in China and providing policy suggestions, so as to expand the application of the ML algorithm in economics.

The paper is organized as follows. The second section introduces the research methods of this paper, including the BP neural network algorithm combined with the DEA model to measure IG and a nest of ML algorithms to measure the drivers of IG. The third section reveals the characteristics of Chinese urban IG and lists the explanatory variables of IG through literature review. In Section 4, firstly, the determinants of IG are calculated by the ML model. Then, the heterogeneity test and robustness test are carried out. The fifth section summarizes the research conclusions and puts forward some policy suggestions.

The article "Evaluating the Performance of Inclusive Growth Based on the BP Neural Network and Machine Learning Approach" was published in 2022. Journal: Comput Intell Neurosci.

## 2. Methodology

In this section, the BP neural network and a nest of ML algorithms used in this paper are introduced in 2.1. Then, a nest of ML used to explore the drivers of IG will be elaborated in 2.2.

### 2.1. BP Neural Network Algorithm

The BP neural network is a multilayer feedforward neural network trained according to the error back propagation (BP) algorithm, which is widely used in the fields of finance and engineering technology. A typical BP neural network consists of three layers: an input layer, hidden layers, and an output layer, as shown in Figure 1. The BP neural network has the characteristic of self-learning. Its operation includes forward propagation and back propagation. The BP neural network model used in this paper is solved by function programming in the Matlab environment. Figure 1 is the structure of the BP neural network algorithm.

According to the concept of IG in previous studies [1, 3, 5], we design a framework of China's urban IG evaluation system composed of 3 levels and 15 specific indicators. The target level reflects that the process of pursuing IG should achieve the balance of economic growth, opportunities, and sharing. The criterion layer reflects the different effects of each subsystem on inclusive growth. The indicator layer describes the basic indicators of inclusive growth, as shown in Table 1. The specific steps of the BP neural network to evaluate IG are as follows:

1. Taking the Index set as the input value of the network and using the DEA model to calculate the inclusive growth efficiency (IGE) as the expected output value of the network, the historical samples are formed together. The data generally need normalization preprocessing. Select *m* samples from *n* historical samples as training samples and *N*-*M* samples as verification samples.
2. Determine the network structure and set the parameters.
3. The network is used to simulate the training samples, and the training output vector is restored by inverse normalization. The simulation output and the expected output of the training samples of the network are linearly regressed to test the performance of the network.
4. The network is used to simulate and predict the verification samples, and the predicted output vector is restored by inverse normalization. Judge whether the error between the simulation predicted output and the expected output of the verification sample of the network meets the requirements, and test the generalization performance of the network.
5. If the error meets the requirements and passes the verification, it indicates that the network has a strong generalization ability and can be used for future prediction. The predicted value can be obtained by inputting a new value. Otherwise, the network is reconstructed by adjusting the training samples and parameter settings for training and verification until satisfactory.

The article "Evaluating the Performance of Inclusive Growth Based on the BP Neural Network and Machine Learning Approach" was published in 2022. Journal: Comput Intell Neurosci.

#### 2.1.1. Calculate the Desirable Output Value of the BP Neural Network

Referring to Sun et al. [28] and Xu et al. [29], we employ the data envelopment analysis (DEA) model to measure urban IG as the expected output value of the BP neural network in China during the statistical period, which is one of the most important methods for efficiency estimation; it comprehensively evaluates the object from the perspectives of input and output, and is more reasonable and scientific than the methods that simply consider the output, such as the principal component analysis and entropy weight method [30]. Previous studies have applied the DEA model to evaluate efficiency, such as energy efficiency, the economic efficiency, innovation efficiency, environmental efficiency, and so on [31, 32]. Tone and Tsutsui [33] proposed an epsilon-based measure (EBM) model, which not only considers the radial proportion of the input frontier value and the actual value, but also reflects the differentiated non-radial relaxation variables among various input factors, effectively improving the accuracy and scientific nature of the results. On this basis, this paper integrates the super-efficiency DEA model proposed by Andersen and Petersen [34] to measure the IGE of sample cities in China.

Assuming that the production system has *n* decision units, each decision unit has three vectors, including input *X*, desirable output *Y*^*g*^, and undesirable output *Y*^*b*^, whose elements can be expressed as *x* ∈ *R*^*m*^, *y*^*g*^ ∈ *R*^*s*^ 1, and *y*^*b*^ ∈ *R*^*s*^ 2; we define matrix *X*, *Y*^*g*^, and *Y*^*b*^ as *X*=[*x*_1_,…, *x*_*n*_] ∈ *R*^*m*×*n*^, *Y*^*g*^=[*y*_1_^*g*^,…, *y*_*n*_^*g*^] ∈ *R*^*s*^1^×*n*^, and *Y*^*b*^=[*y*_1_^*b*^,…, *y*_*n*_^*b*^] ∈ *R*^*s*^2^×*n*^, where *x*_*i*_ > 0, *y*_*i*_^*g*^ > 0, and *y*_*i*_^*b*^ > 0(*i*=1,2,…, *n*). The SBM-DEA model to evaluate the efficiency is expressed as:

(1) $$\begin{array}{c} \sigma =\begin{array}{cc} \min & \frac{1-\left(1/m\right)\sum_{i=1}^{m}s_{i}^{-}/x_{i0}}{1+\left(1/s_{1}+s_{2}\right)\left(\sum_{r=1}^{s_{i}}s_{r}^{g}/y_{r0}^{g}\right)+\left(\sum_{r=1}^{s_{2}}s_{r}^{b}/y_{r0}^{b}\right)},\\ \text{st} & \left\{\begin{array}{c} x_{0}=X\lambda +s^{-},\\ y_{0}^{g}=Y^{g}\lambda -s^{g},\\ y_{0}^{b}=Y^{b}\lambda -s^{b},\\ s^{-}\geq 0,s^{g}\geq 0,s^{b}\geq 0,\lambda \geq 0, \end{array}\right. \end{array} \end{array}$$

where *s*^−^, *s*^*g*^, and *s*^*b*^ represent the input, the desirable output, and the undesirable output, respectively; the weight vector is *λ* . The objective function *σ* is strictly monotonically decreasing with respect to *s*^−^, *s*^*g*^, and *s*^*b*^ as well as 0 ≤ *σ* ≤ 1. When *σ*=1, *s*^−^ = 0, *s*^*g*^ = 0, and *s*^*b*^ = 0, it indicates that the decision-making unit (DMU) is in the effective status. When *σ*＜1, it means that there is redundancy in the DMU, and the efficiency can be improved by optimizing the configuration.

The article "Evaluating the Performance of Inclusive Growth Based on the BP Neural Network and Machine Learning Approach" was published in 2022. Journal: Comput Intell Neurosci.

According to the conceptual framework of IG in previous studies [35–38], an economy not only pursues economic growth, but also provides fair employment and education opportunities. In addition, the performance of economic growth can be fairly distributed among social members. Thus, it is indispensable to establish a comprehensive indicator for evaluating it, as well as fully consider the impact of IG inputs, desirable IG outputs, and undesirable IG outputs. This study selected an indicator to represent these inputs and outputs in the following way:

1. Inputs: Referring to Sun et al. [28], economic system runs need labor and capital. For this consideration, we use the total number of regional employees and private enterprises owners at the end of each year as the corresponding proxy variable.
2. Desirable outputs: For developing countries, an essential prerequisite for IG is economic growth, while providing access to education and healthcare for social members. Therefore, we select the GDP, the ratio of teachers to students in basic education, and the number of medical personnel per thousand population to represent the desired outputs of economic growth, equal access to education, and equal social security, respectively. Considering the particularity of the DEA model, we use the entropy weight method to synthesize a desirable output index.
3. Undesirable outputs: IG also emphasizes equal opportunities to participate in employment and equitable income distribution. Thus, the registered urban unemployment rate is selected as an undesirable output. In addition, since China's income gap is mainly reflected in the urban-rural income gap, the urban-rural income ratio is also regarded as an undesirable output to income distribution. Similarly, these indicators are synthesized an undesirable output index.

The article "Evaluating the Performance of Inclusive Growth Based on the BP Neural Network and Machine Learning Approach" was published in 2022. Journal: Comput Intell Neurosci.

#### 2.1.2. Determination of the BP Neural Network Structure

1. Enter the number of layer nodes: The number of nodes in the input layer is determined by the input index. The evaluation index *r* is 15, and thus the number of nodes in the input layer is 15.
2. Network hidden layers: Since any continuous function in the closed interval can be approximated by a hidden layer BP neural network, a three-layer BP network can complete any n-dimensional to m-dimensional mapping. Thus, we choose a single-layer hidden layer network.
3. Number of hidden layer nodes: Through comparative training under different hidden layer nodes, the number of hidden layer nodes is finally determined to be 14.
4. Number of output layer nodes: In the training stage of the BP neural network, the expected output value of the sample is a known quantity. In this paper, it is the comprehensive score of each year, and thus the number of nodes in the output layer is 1.
5. We conducted data shuffle and 50% cross-validation to make the model more robust. Specifically, we divide the data into five equal parts. Each experiment uses one piece of data for testing, and the rest is used for training. After 5 times process, we calculate the average value.

#### 2.1.3. Parameter Setting of the BP Neural Network

1. Training function: In the training of the BP neural network, the data within the training sample range can be well fitted. For the data outside the training sample range, if the fitting degree is good, it is said that it has a strong generalization ability and strong prediction ability for unknown data. The generalization ability actually reflects the ability of the BP neural network to identify new sample sets outside the training sample set, which plays a decisive role in whether the BP neural network can be applied in practice. The conventional method to enhance the generalization ability is to call the trainbr function, and thus the trainbr function is selected to train the network.
2. Expected error (goal): The expected error value is finally determined as 0.0001 through training.
3. Learning step length (LR): The learning step determines the weight change generated in each cyclic training. The selection range of the learning step is generally between 0.02 and 0.7. Through training, the final learning step is 0.02.
4. Maximum learning steps (epochs): Through comparative training under different maximum learning steps, the maximum learning steps are finally determined to be 150.
5. Momentum factor (MC): Through comparative training under different momentum factors, the momentum factor is finally determined to be 0.80.
6. To employ the traingdm algorithm to train the BP net, the main code for Matlab is as: [net, tr] = train (net, P', T);

The article "Evaluating the Performance of Inclusive Growth Based on the BP Neural Network and Machine Learning Approach" was published in 2022. Journal: Comput Intell Neurosci.

### 2.2. Machine Learning Algorithms

#### 2.2.1. Random Forest Algorithm

The RF algorithm has a long reputation in solving classification problems. In recent years, it has been widely used in many interdisciplinary fields, such as finance [39], environmental protection [40, 41], and marketing [42, 43]. It is based on a set of trees, and the measurement is the average projection's mean value obtained at the end of each tree, eliminating the lack of robustness of individual single trees [27]. Each tree is produced using a randomly selected subset of independent variables. The estimation model can be expressed as:

(2) $$\begin{array}{c} \hat{Y}=\frac{1}{q}\sum_{i=1}^{q}g\left[k\left(x\right)\right]. \end{array}$$

Here, *g*(*x*) is a set of kth learner random trees and *x* is the vector of the input features. The RF's final estimation is the average of all the outcomes of each tree. Therefore, each individual tree affects the RF estimation at such weights [27]. It is superior to other ML algorithms since it can automatically receive training data from subsets and trees using random algorithms [44].

#### 2.2.2. XGBoost Algorithm

The XGBoost algorithm is an integrated learning model, which has improved the CART regression tree model [45]. The idea of this algorithm is to continuously add trees, and the newly added trees will split and grow another tree according to the features. The process of adding trees is learning new functions. Drop each tree onto the corresponding leaf node according to the sample characteristics, and add the scores on each leaf node to get the predicted value [46]. Its estimation function is:

(3) $$\begin{array}{c} \hat{Y}=\vartheta \left(x_{i}\right)=\sum_{k=1}^{K}f_{k}\left(x_{i}\right),\\ F=\left\{f\left(x\right)=w_{q\left(x\right)}\right\}\left(q:R^{m}⟶T,w\in R^{T}\right). \end{array}$$

In the function, *w*_*q*(*x*)_ is the score of leaf node *q*; *f*(*x*) is one of the regression trees; and *T* represents the number of leaf nodes. As an additional advantage, the XGBoost is not influenced by multicollinearity [47]. To avoid excessive fitting or inadequate fitting, several parameters need to be adjusted before using the model, as to improve the model's performance.

#### 2.2.3. CatBoost Algorithm

The CatBoost is a novel version of the gradient-boosting decision tree algorithm. It has powerful learning capabilities to manage extremely nonlinear data [27]. The main feature is that it can efficiently and reasonably deal with category features and gradient deviation, and predict migration problems, so as to improve the accuracy and the generalization ability of the algorithm [48].

The article "Evaluating the Performance of Inclusive Growth Based on the BP Neural Network and Machine Learning Approach" was published in 2022. Journal: Comput Intell Neurosci.

The predicted function is described as follows:

(4) $$\begin{array}{c} g^{t}=\arg\min\frac{1}{M}{\sum \left(-f^{t}\left(X_{k},Y_{k}\right)-g\left(X_{k}\right)\right)}^{2}. \end{array}$$

In this function, *g*(*X*) represents the decision tree function, while the gradient's conditional distribution is expressed as *f*^*t*^(*X*_*k*_, *Y*_*k*_).

#### 2.2.4. LightGBM Algorithm

LightGBM is an efficient implementation of XGBoost. Its idea is to discretize continuous floating-point features into k discrete values and construct a histogram with a width of k. Then, traverse the training data and calculate the cumulative statistics of each discrete value in the histogram. In feature selection, we only need to traverse to find the optimal segmentation point according to the discrete value of the histogram. In addition, the use of leaf wire strategy with depth limit saves a lot of time and space consumption [49, 50]. LightGBM incorporates many T regress tress ∑_*t*=1_^*T*^*g*_*t*_ (*X*) to estimate the final model which may be expressed as follows:

(5) $$\begin{array}{c} \hat{Y}=\sum_{t=1}^{T}g_{t}\left(X\right), \end{array}$$

where the regress trees may be expressed as *W*_*p*(*x*)_, and *p* ∈ {1,2,…, *N*}. The number of tree leaves is represented as *N*; *p* means the trees' decision rule; and the sample weights of the leaf nodes are expressed as *w*.

## 3. Characteristics of IG and Plausible Explanatory Variables for IG

In this section, we mainly report the time trend characteristics of the urban IGE in China, which is calculated by the DEA model in 3.1. Then, 10 plausible explanatory variables for urban IG will be selected by combing the existing literature introduced in part 3.2.

### 3.1. Characteristics of IG

Figure 2 revealed the time trend characteristics of the mean value of IGE calculated based on the DEA method. It shows that the IGE of cities showed a gradual upward trend during the statistical period. However, the growth rate in 2008 and 2010 was relatively low, and may be due to the negative impact of the global subprime mortgage crisis in these years. It is worth noting that the IGE shows stable growth after 2016, which may be due to China's economy entering the new normal period and paying more attention to the high-quality growth of the balance between the economic system and the social system. Figure 2 is the trend of the IGE in China during 2005–2020.

### 3.2. Plausible Explanatory Variables for Inclusive Growth

This study uses a list of explanatory variables, and the selection of these variables is mainly based on the existing empirical literature. Specifically, it includes economic growth, financial development, digitization, foreign direct investment, government intervention, the urbanization process, entrepreneurship, innovation, urban size, and industrial structure. Next, we briefly describe the proxy of each variable, and will build a relationship thermodynamic diagram based on the data of these variables, as shown in Figure 3, as well as statistical description in Table 2.

The article "Evaluating the Performance of Inclusive Growth Based on the BP Neural Network and Machine Learning Approach" was published in 2022. Journal: Comput Intell Neurosci.

#### 3.2.1. Economic Growth

The impact of economic growth on IG is debatable. In Kuznets' hypothesis [51], inequality must rise in the early stages of economic development, but falls after a certain point of economic development. However, the pattern has changed in recent decades, with income inequality not only in developing countries but also in OECD countries [52]. Thus, we employ GDP per capita (pgdp) to reflect the urban economic growth, which describes an area's economic and financial resources and how efficiently they are allocated [53, 54], and detect its impact on urban IG.

#### 3.2.2. Financial Development

Referring to [55], better functioning financial systems foster economic growth and poverty alleviation; moreover, a more equitable distribution of economic opportunities enhances overall economic development. Thus, financial development (fd) may play an important role in accomplishing IG. Based on this, this paper selects the ratio of the balance of deposits and loans to the GDP of the region to represent the financial development level of the cities.

#### 3.2.3. Digitization

The advent of the digital age has injected vitality into the economy, especially in remote areas and poor groups [56, 57]. These groups could accomplish self-employment and increase their income through digital platforms. In addition, people can enjoy such services as telemedicine, distance education, and digital finance through the Internet. Therefore, digitization may promote IG, and thus we choose the Internet penetration rate (inter) of cities to represent the urban digitalization level.

#### 3.2.4. Foreign Direct Investment

Previous studies have confirmed the positive impact of foreign direct investment (fdi) on the host country, such as introducing more advanced technology and knowledge, promoting regional employment, and so on [58, 59]. Foreign direct investment is especially well suited to effecting cross-border adoption transfer and translating it into broad-based growth, not least by upgrading human capital [60]. We choose the actual utilization amount of foreign direct investment in the city to take the right number to represent its development level.

The article "Evaluating the Performance of Inclusive Growth Based on the BP Neural Network and Machine Learning Approach" was published in 2022. Journal: Comput Intell Neurosci.

#### 3.2.5. Government Intervention

Several studies have proved that government expenditure provides better educational opportunities for school-age students in poor areas; hence, it improves local human capital and alleviates poverty [61]. Furthermore, if the government increases its investment in infrastructure, it will improve the employment rate and prosper the regional economy [62]. In addition, policies conducive to agriculture can increase the income of rural residents [63]. Therefore, we use the ratio of Urban Fiscal Expenditure to regional GDP as a proxy for government intervention (gove).

#### 3.2.6. Urbanization Process

As the largest developing country in the world, China's urbanization rate has reached about 58% by 2016, higher than the average level of the world and Asia [64]. Then, too fast urbanization and extensive planning tend to increase the gap between the rich and the poor, increase unemployment, and bring too high house prices [65, 66], which may hinder the realization of IG. Therefore, we use the ratio of urban house investment to GDP (house) to represent urbanization.

#### 3.2.7. Entrepreneurship

Previous studies have confirmed the positive impact of entrepreneurship [15], especially female entrepreneurship [67, 68], on inclusive economic growth. The process of entrepreneurship can not only increase the income of entrepreneurs and reduce poverty, but it also provides employment opportunities and reduces the unemployment rate. Therefore, we choose the number of newly increased private enterprises registered in the industrial and commercial authorities in the city every year as the proxy variable of entrepreneurship (enterp).

#### 3.2.8. Innovation

Innovation implies the introduction of new technologies, management models, or products into the economic system, which can bring about the improvement of production efficiency and social progress [69]. Thus, it may have a potential impact on growth inclusiveness. Ivanic and Martin [70] examined the implications of productivity improvements in agriculture, industry, and services for global poverty and concluded that in poor countries, increases in productivity generally have a poverty-reduction effect. Based on this, this paper selects the number of patent invention applications in the city as the agent variable of innovation (innovation).

#### 3.2.9. Urban Size

Based on China's current situation, different urban sizes lead to different economic agglomeration and industrial development [71]. Large cities often have good resource endowments and location advantages, and macro-control policies tend to sustainable development [72]; thus, they may show a higher level of IG. Therefore, we choose the logarithm of urban population to represent the size of the city and study its impact on urban IG in China.

The article "Evaluating the Performance of Inclusive Growth Based on the BP Neural Network and Machine Learning Approach" was published in 2022. Journal: Comput Intell Neurosci.

#### 3.2.10. Industrial Structure

In developing countries, a large population employed in the agricultural sector usually means a large number of low-income groups. Therefore, improving the level of industrialization is the performance of industrial structure optimization. Moshi [73] built a case for the imperative of boosting the manufacturing sector as the surest way of tackling Africa's development challenges of fragile economic growth, poverty, inequality, and vulnerability to socio-economic shocks. Therefore, we calculate the proportion of the added value of the secondary industry and the tertiary industry in GDP as the proxy variable of the industrial structure (ind).

### 3.3. Descriptive Statistics of the Explanatory Variables

The data used in this study are mainly from China Urban Statistical Yearbook, China Rural Yearbook, and government official statistical websites. To ensure the reliability of the data, we checked the data and deleted the cities with serious data deficiency. The final research sample was 281 prefecture-level cities and cities above the prefecture level in China from 2005 to 2020. Figure 3 presents the thermodynamic diagram among independent variables.

Due to the specific conditions of different countries, the conclusions of the previous studies on the above explanatory variables may not be applicable to Chinese cities. Therefore, it is very necessary to deeply explore whether and to what extent the above factors contribute to China's urban IG. This is the focus of the next section of this paper. Table 2 is the statistics summary of the variables.

## 4. Determinants of Inclusive Growth

In this section, we focus on exploring the determinants of IG in China. We mainly use a series of ML algorithms for calculation, and the process is stated in 4.1. The determinants of IG in China are calculated by the ML method in 4.2. In 4.3, we mainly conducted the heterogeneity test. In addition, we introduce the robustness test to verify the robustness of the results of the ML algorithm.

### 4.1. Machine Learning Modelling

#### 4.1.1. ML Modelling Steps

The process of determining the driving factors of IGE by the ML method includes data preprocessing, model construction, model prediction, and analysis. The specific steps are as follows:

*(1) Step One: Data Preprocessing*. We first normalize the data and then conduct ML training and learning. The normalization formula is:

(6) $$\begin{array}{c} \mu =\frac{x-x_{\min}}{x_{\max}-x_{\min}}, \end{array}$$

where *μ* represents the data after normalization while *x* means the data before normalization; *x*_min_ and *x*_max_ denote the largest and the smallest data, respectively. After normalization, we divide the dataset into a training set and a testing set, and the weight is 70% and 30%, respectively.

*(2) Step Two: Model Building*. We select a nest of algorithms including the Random forest, XGBoost, CatBoost, and LightGBM algorithms to build the ML model. Firstly, based on the characteristics of each algorithm, the initial parameters of the algorithm are set. Next, set the adjustment parameters and parameter selection range, referring to [74]; we use the 10-fold cross-method to select the parameters and evaluate the results based on the correlation coefficient between the measured value and the predicted value. Finally, the optimal parameters of the model are obtained, and then the training set is used for model training, so as to save the optimal model.

*(3) Step Three: Prediction and Analysis*. We input the test set data into the ML models, respectively, and output the prediction results. Then, the measured value and the predicted value of the model are mathematically analyzed, and the prediction ability of the model is compared according to the model evaluation method. At the same time, the size of the model is analyzed according to the construction time of the model.

The article "Evaluating the Performance of Inclusive Growth Based on the BP Neural Network and Machine Learning Approach" was published in 2022. Journal: Comput Intell Neurosci.

#### 4.1.2. Model Evaluation Method

In this study, goodness of fit (*R*^2^), mean square deviation (RMSE), mean absolute error (MAE), and mean absolute percentage error (MAPE) are used to evaluate the model. Among them, *R*^2^ compared the predicted value with the mean value only, and the closer its result was to 1, the higher the accuracy of the ML model. The smaller the value of other indicators, the higher the accuracy of the model. The calculation methods of each index are as follows:

(7) $$\begin{array}{c} R^{2}=\frac{{\left(\sum_{i=1}^{n}\left(yo_{t}-\bar{y}o\right)*\left(ym_{t}-\bar{y}m\right)\right)}^{2}}{\sum_{t=1}^{n}{\left(yo_{t}-\bar{y}o\right)}^{2}*\sum_{t=1}^{n}{\left(ym_{t}-\bar{y}m\right)}^{2}},\\ \text{RMSE}=\sqrt{\frac{1}{n}\sum_{t=1}^{n}{\left(yo_{t}-ym_{t}\right)}^{2}},\\ \text{MAE}=\frac{1}{n}\sum_{i=1}^{n}\left|\left(yo_{t}-ym_{t}\right)\right|,\\ \text{MAPE}=\sum_{t=1}^{n}\left|\frac{yo_{t}-ym_{t}}{yo_{t}}\right|*\frac{100}{n}. \end{array}$$

where *n* means the number of data; *ym* is the predicted result; *yo* is the real value; and $\bar{y}m$ and $\bar{y}0$ denote the mean value of the predictive result and the real result, respectively.

#### 4.1.3. ML Model Parameter Setting

During the construction of each ML model, the initial value of parameters is set based on the algorithm characteristics of different models and the experience of parameter adjustment. In this process, refer to the Gridsearch method provided by Bergstra and Bengio [75]. Then, the best parameters of each model are obtained according to the evaluation index, and the best parameters and the training set are used to construct each machine learning model. Then, the trained model is used for IGE driver evaluation. The parameter settings of each model are shown inTables 3 and 4.

The article "Evaluating the Performance of Inclusive Growth Based on the BP Neural Network and Machine Learning Approach" was published in 2022. Journal: Comput Intell Neurosci.

### 4.2. Determinants of Inclusive Growth

We input the test set into each model for calculation. The comparison between the predicted results of ML and the actual results is shown in Figure 4. A significant advantage of the ML algorithm is that it can automatically calculate the important percentage of the contribution of different drivers to IGE. Meanwhile, these ML methods do not assume that there is a linear relationship between the 10 explanatory variables and IGE. However, the results of different models are different, as shown in Figure 5. Among the determinants calculated by the RF algorithm, the innovation contribution weight is the largest, more than 65%; XGBoost's results show that the contribution of entrepreneurship and innovation is roughly the same, accounting for about 35% each. Among the results of the CatBoost algorithm, innovation contributes the most, accounting for about 32%. Finally, in the results of the LightGBM algorithm, the contribution of city size and economic growth is in the forefront. Therefore, it is essential to determine the optimal model and obtain the results according to the optimal model. The performance evaluation of each model is shown in Table 5.

Table 5 reveals the performance of the different ML algorithms. From goodness of fit *R*^2^, we can see that the goodness of fit of the XGBoost algorithm is 0.995, which is closest to 1 and the largest among all ML models. By comparing the MAE and MAPE, we can see that the MAE value of the training set and the test set of the XGBoost algorithm is 0.03, which is the smallest among all the algorithms. For MAPE, the XGBoost algorithm also has the smallest value, which shows that the ML model based on the XGBoost algorithm is the best model for the study of IGE determinants in this paper. Furthermore, the comparison between the prediction results of different algorithms presented in Figure 4 and the real value also verifies that the prediction value of XGBoost is closest to the real value. Therefore, next, we mainly analyze the operation results based on the XGBoost model. Figure 4 illustrates the comparison of the ML-predicted value and the real value.

Based on the above selection process of the optimal ML model, we mainly focus on Figure 5(b), which is the calculation result of the ML model established based on the XGBoost algorithm. This figure shows that among the 10 explanatory variables we selected for IGE, entrepreneurship and innovation contribute the most, accounting for about 35%, respectively. It shows that for the sample cities in the statistical period, entrepreneurship and innovation are the core factors driving urban IG, which is consistent with the previous research conclusions [67–70]. The possible reason is that these factors can drive the improvement of production efficiency, so as to promote the survival and development of small- and medium-sized enterprises (SMEs) and bring better employment opportunities. At the same time, innovation leads to new technologies and inventions, so as to benefit more members of society. These are followed by financial development, which contributes about 8%. The possible reason is providing financial support for enterprises and helping SMEs solve their financing difficulties; thus, its role cannot be underestimated. Then comes economic growth, which contributes about 7%. It shows that for developing countries such as China, the contribution of economic growth to IG is relatively small relative to innovation and entrepreneurship, and simply pursuing the economic growth model of regional GDP is not necessarily of great value to IG. Next, is the city size, which contributes about 6%, which also verifies that large cities may play an economic agglomeration effect and contribute to IG. This is followed by the industrial structure, whose contribution is about 5%, indicating that industrialization can narrow the income gap and benefit the poor to a certain extent, but its role is limited. Then, there is the process of urbanization, whose contribution is about 4.5%, followed by digitization and foreign direct investment. The proportion of government intervention is the least, whose contribution is about 2%. It shows that in current China, the government has not played its due role in promoting fair opportunities and narrowing the gap between the rich and the poor.

The article "Evaluating the Performance of Inclusive Growth Based on the BP Neural Network and Machine Learning Approach" was published in 2022. Journal: Comput Intell Neurosci.

### 4.3. Heterogeneity Test

To further capture the differences of IGE determinants in geographic distribution, region-based heterogeneity tests were performed. Firstly, we divide all sample cities into three regions, namely eastern, central, and western regions, according to different locations. Similarly, the level of economic development of the cities in the three regions of China declines in turn. Then, we employ the XGBoost algorithm to build a ML model to explore the influence of independent variables on dependent variables and the importance of each variable in the above three regions, and try to prove whether the determinants of different regions will change.  Figure 6 reports the experimental results and Figure 7 shows the dynamic fitting level between the real value and the predicted value; Table 6 shows the evaluation of XGBoost performance based on the heterogeneity test. Figure 7 is the contribution of the determinants of different regions to IGE.

The three subparagraphs in Figure 6 reveal the experimental results of the eastern, central, and western regions in China, respectively. Overall, among the factors that determine urban IGE in different regions, economic growth and innovation contribute the most weight, and the importance ranking of other determinants has changed, compared to the results of the total sample cities. Specifically, for cities in the eastern region, the contribution of economic growth to IGE is the largest, accounting for about 50%. The calculations for this region support Kuznets' hypothesis that economic growth to a certain extent can reduce social income disparities and inequality [51]. Benefits from the favorable business environment and advantages in geographical resources, the eastern region leads China in economic development. For example, the three rivers of the Yangtze River and the Pearl River Delta have formed a good economic agglomeration and spillover effect to the surrounding cities. In the second and third places are innovation and entrepreneurship, respectively; therefore, innovation and entrepreneurship form a joint force to narrow the income gap and boost the realization of IGE in the eastern region. However, the role of other factors to promote IGE is not very obvious in this region.

Next, for the cities in the central region, the biggest contribution to driving IGE is innovation, while the second most decisive IGE factor is foreign direct investment, followed by economic growth that ranks third, and the impact of other factors is not obvious. It may be that some cities in Central China are usually engaged in backward industries, such as bottom manufacturing, and some are resource-based cities, such as coal cities. These industries have low production capacity and low added value. Thus, innovation is essential to drive local industrial transformation and urban economic upgrading. In addition, after the introduction of foreign investment, it can introduce foreign advanced technology, management experience, and talents into domestic enterprises, help enterprises improve business performance, inject fresh blood into the economic growth of these cities, as well as increase people's income by providing employment opportunities in these foreign enterprises and promote urban IG. Therefore, the power of foreign direct investment in driving IGE in the central region should not be underestimated.

The article "Evaluating the Performance of Inclusive Growth Based on the BP Neural Network and Machine Learning Approach" was published in 2022. Journal: Comput Intell Neurosci.

Further, through Figure 6(c), we analyze the ranking changes of the determinants affecting IGE in cities in western China. It is worth noting that in the western region, similar to cities in the central region, innovation still contributes the most to the improvement of urban IGE, with 53% more. At the same time, the contribution of other influencing factors to IGE has also changed, which is obviously different from the other two regions. Specifically, foreign direct investment ranked second, with a contribution of about 25% to IGE, which is more important than the eastern region. The possible reason is that the economy of western China is the most backward, and the marginal contribution of introducing foreign capital is more significant than that of other regions. This is followed by entrepreneurship, which contributes about 10% to IGE. The digital level contributes to IGE, followed by financial development and industrial structure. Other factors have little impact. This implies that the western region has weaknesses in finance development, technology innovation, industry structure, and many other aspects; hence, the number of factors determining IGE is more than that in other regions, and improvement and efforts need to be made in many aspects.  Figure 8 is the comparison of the ML-predicted value and the real value in different regions.

Finally, from the comparison between the predicted value and the real value of the XGBoost algorithm in the different regions revealed in Figure 7, it can be seen that our regional heterogeneity test results have high accuracy, and the predicted results completely coincide with the real value. In addition, the performance of the ML model reported in Table 5 also demonstrates the reliability of the heterogeneity test's conclusion in this paper. As can be seen from Table 6, the *R*^2^ of the XGBoost algorithm in the three regions is 1, indicating that the results of ML are the real result. The results of machine learning based on different regions are even better than those based on all the samples.

### 4.4. Robust Test

In order to further verify that the conclusion obtained by the XGBoost algorithm is robust and reliable, we mainly employ two methods of the robustness test. First, the GBDT algorithm is introduced to verify XGBoost results. The advantage of this algorithm is that it can deal with nonlinear data and is flexible [76–78]. In addition, it uses some robust loss functions, such as the Huber loss function and the Quantile loss function, which are very robust to outliers. Second, we use the traditional econometric model to regress and compare the calculation results with the ML model.

The article "Evaluating the Performance of Inclusive Growth Based on the BP Neural Network and Machine Learning Approach" was published in 2022. Journal: Comput Intell Neurosci.

#### 4.4.1. GBDT Algorithm

GBDT is a gradient lifting decision tree. Its output results are accumulated from several decision trees contained in it. Each decision tree is a fitting of the combined prediction residuals of the previous decision trees and a “correction” to the results of the previous model. It trains a set of CART regression trees serially, and finally sums up the prediction results of all regression trees to obtain a strong learner. Each new tree fits the negative gradient direction of the current loss function. Finally, the summation of this set of regression trees is output to obtain the regression result. The parameters we set are: number of base learners = {100}; learning rate = {0.1}; maximum depth of tree = {10}; and threshold of node partition impurity = {0}. The performance evaluation of the model is shown in Table 7. The calculation results and the comparison between the predicted value and the real value are shown in Figure 8.

From the model performance evaluation in Table 7, the performance of GBDT is second only to XGBoost; the accuracy of its calculation results is high and is superior to the RF, Catboost, and LightGBM algorithms. Among the determinants of IGE revealed in Figure 8(a), entrepreneurship and innovation still contribute the highest degree of importance, with a total of about 70%, while the calculation results of other factors change slightly compared with XGBoost. This shows that the results calculated by the XGBoost algorithm in this paper are robust.

#### 4.4.2. Econometric Model Regression

We further introduce the traditional econometric method to verify the research results of the ML model. In the setting of regression model, the independent variable is an explanatory variable, and the dependent variable is IGE which is measured by the DEA model.  Table 8 reports the regression results and *R*^2^ of the econometric model. Among them, the regression result of the first column is the regression result of controlling the fixed effect of urban individuals by ordinary least squares (OLS). The second column is the regression result that controls the time fixed effect. The third column is the regression results of using the OLS method to control the urban individual and time fixed effects at the same time. The last column is the random effect model estimation.

According to the *R*^2^ of the four econometric models in Table 8, we can see that under the model of controlling the fixed effect of urban individuals and time effect at the same time, the *R*^2^ of the regress result is 0.79533, which is the best result. Therefore, we focus on comparing the results of this column with the calculation results of ML under the previous XGBoost algorithm to judge whether the results of the ML model are robust.

The article "Evaluating the Performance of Inclusive Growth Based on the BP Neural Network and Machine Learning Approach" was published in 2022. Journal: Comput Intell Neurosci.

It can be seen from Table 8 that among all the driving factors of IGE, the variables with a positive coefficient at the 1% significance level are innovation, industrial structure, digitization, entrepreneurship, and economic growth. It is suggested that these factors have the most significant positive driving effect on urban IGE. However,the coefficient of urbanization and foreign direct investment is negative, indicating that these two factors significantly inhibit IGE in Chinese cities. The two driving factors of government intervention and population size are significant at the significance level of 5%, indicating that their importance in influencing IGE in cities is lower than the previous factors. The coefficient of financial development is positive, but not significant. This result is also in line with the conclusion of the XGBoost computational ML algorithm, although there are some subtle differences. However, the econometric model of *R*^2^ is only 0.79533, which is far lower than the goodness of fit of the ML algorithm, 0.995. The possible reason for the difference is that the econometric model assumes the linear relationship between independent variables and dependent variables, while the ML model calculates the nonlinear relationship; thus, the latter is more consistent with the real situation and more robust and superior than the traditional method.

## 5. Conclusion and Policy Suggestion

### 5.1. Conclusion

With China's economic development entering the new normal stage, the pursuit of high-quality development has become China's core strategy. IG has become an important path to realize this strategy. Based on this background, this paper introduces the BP neural network algorithm model to calculate the IGE level of 281 prefecture-level cities and cities above the prefecture level in China from 2005 to 2020. Furthermore, in order to overcome the disadvantages of the potential endogeneity of econometric models, the inability to deal with the multicollinearity of variables, model linearity assumption, and so on, we introduce a nest of ML algorithms to calculate the driving factors of urban IGE in China.

By comparing the results of different algorithms, such as RF, XGBoost, CatBoost, and lightGBM, we find that the calculation performance of the XGBoost algorithm is the best. Among the driving factors of IGE in Chinese cities based on the XGBoost algorithm, the most important driving forces are entrepreneurship and innovation, which contribute 70% of all. The total contribution of other factors is about 30%. Further, we conducted a heterogeneity test based on geographical locations, and divided the sample cities into the East, Central, and West regions. We found that the drivers of urban IGE are different in different regions, and analyzed the possible reasons for the differences in the results. Next, in order to verify the robustness of the previous conclusion, we tested the robustness of the previous conclusion by replacing the ML algorithm with a traditional econometric model, which confirmed the robustness of the previous conclusion and the superior performance of the XGBoost algorithm in calculating the impact of IGE in Chinese cities.

The article "Evaluating the Performance of Inclusive Growth Based on the BP Neural Network and Machine Learning Approach" was published in 2022. Journal: Comput Intell Neurosci.

### 5.2. Policy Suggestion

Based on the importance ranking of the determinants of IGE in Chinese cities calculated by the XGBoost algorithm, and the results of the heterogeneity analysis, we provide the following policy suggestions:

First, at the national level, policy makers should actively promote a “Mass entrepreneurship and innovation” strategy. On the one hand, we should promote urban innovation and entrepreneurship as a long-term development strategy. Specifically, it is essential to create a business environment conducive to entrepreneurship, and give entrepreneurs and innovative individuals incentives such as tax concessions and subsidies, as well as financial and technology support. On the other hand, a convenient communication network and collaboration mechanisms should be formed between urban scientific research institutions, universities, the government, and enterprises to promote the effective transformation of scientific research achievements into the driving force of urban entrepreneurship and innovation to further promote the IGE of the city.

Secondly, cities in different regions should promote their IGE level based on their own characteristic location comparative advantage. For the eastern region, its successful development experience should be shared with the central and western regions to form an interactive mechanism of knowledge and experience by the digital platform. For the central and western regions, they should develop characteristic industries based on their own features, and gradually eliminate backward production capacity and develop advanced industries. To further attract capital and talents, they should ensure the local people get rid of relative poverty and increase social welfare, so as to promote the coordinated linkage of urban IGE. In addition, they should increase the process of new infrastructure, introduce advanced digital infrastructure such as 5G, Internet of things, and artificial intelligence, and promote urban development through digital transformation.

The article "Evaluating the Performance of Inclusive Growth Based on the BP Neural Network and Machine Learning Approach" was published in 2022. Journal: Comput Intell Neurosci.

Finally, the prerequisite for innovation and entrepreneurship is the supply of talents. Therefore, the state should pay attention to the cultivation of scientific and technological talents and entrepreneurs. For example, set up entrepreneurship-related training courses in universities to closely connect theory and implementation. Schools should pay attention to cultivating students' innovative thinking, rather than pursuing the so-called high score. For the policy-making institutions in each city, especially in areas with backward IGE level, policies should be formulated to attract talents and actively introduce high-quality human resources, so as to realize innovation and entrepreneurship based on human capital and promote the development of IGE.

### 5.3. Limitations and Future Research

Limited by the scope of our research, this paper inevitably has the following limitations:

Firstly, because there is no consistent view on the concept and measurement of IG in the academic field, this study is only based on the existing literature to measure the inclusive growth efficiency of Chinese cities. Future research needs to try a variety of different methods, build a more complex comprehensive index system to measure inclusive growth, expand the range of data samples, such as research based on international inclusive growth and inclusive growth in the Asia Pacific region, and enrich academic contributions.

Secondly, due to the availability of data, this study only combs 10 drivers of inclusive growth according to the existing literature. There may be some other potential factors in reality, but they are not taken into account. Therefore, future research will further explore the impact and contribution of other factors in order to find more drivers of inclusive growth.

Finally, although the machine learning method has good accuracy and performance in measuring the inclusive growth of Chinese cities, the potential “black box” problem makes us unable to further explore the intermediary mechanism and the spatial spillover effect of influence. Therefore, in the future, we will try to cooperate with the most cutting-edge machine learning methods and spatial econometric models to deeply explore the spatial effect as well as the mechanism of these factors driving inclusive growth.

## Figures and Tables

**Figure 1:** The structure of the BP neural network algorithm.

**Figure 2:** The trend of the IGE in China during 2005–2020.

**Figure 3:** The thermodynamic diagram among independent variables.

**Figure 4:** The comparison of the ML-predicted value and the real value. (a) RF, (b) XGBoost, (c) CatBoost, and (d) LightBGM.

The article "Evaluating the Performance of Inclusive Growth Based on the BP Neural Network and Machine Learning Approach" was published in 2022. Journal: Comput Intell Neurosci.

**Figure 5:** The contribution of the determinants for IGE. (a) The result from the RF algorithm, (b) the result from the XGBoost algorithm, (c) the result from the CatBoost algorithm, and (d) the result from the LightGBM algorithm.

**Figure 6:** Contribution of the determinants of different regions to IGE. (a) Eastern region, (b) central region, and (c) western region.

**Figure 7:** The comparison of the ML-predicted value and the real value in different regions. (a) Eastern region, (b) central region, and (c) western region.

**Figure 8:** The results of the GBDT algorithm. (a) The result from the GBDT algorithm; (b) the comparison between the real and predicted values.

**Table 1:** Measurement system of the inclusive growth level in China.

Target layer	Rule layer	Index layer	Positive\negative effect	Unit
Economic growth	Economic growth rate	X1 per capita GDP	+	Yuan/person
		X2 annual GDP growth rate	+	%
	Economic growth efficiency	X3 labor productivity	+	
		X4 capital productivity	+	
		X5 total retail sales of consumption goods per capita	+	Yuan
Fairness of opportunities	Employment opportunities	X6 proportion of employed population in secondary and tertiary industries	+	%
		X7 urban unemployment rate	−	%
	Educational opportunities	X8 ratio of students in primary schools	+	%
		X9 ratio of students in middle schools	+	%
	Medical opportunities	X10 number of health technicians	+	Per thousand population
		X11 number of medical institutions	+	Per thousand population
Achievement sharing	Income distribute	X12 rural per capita net income	+	Yuan/person
		X13 per capita disposable income of urban residents	+	Yuan/person
		X14 per capita income ratio of urban and rural residents	−	Multiple
		X15 proportion of labor wage in GDP	+	%

**Table 2:** The statistics summary of the variables.

Variable	Obs	Mean	Std.Dev.	Min	Max
IGE	4,496	0.374	0.0669	0.237	1.029
pgdp	4,496	53706	34539	6457	467749
fd	4,496	3.650	8.806	0.00917	98.29
fdi	4,496	4.329	0.852	0.477	6.489
Gove	4,496	0.335	0.640	0.00241	1.871
Inter	4,496	0.227	0.153	0.00347	0.870
Lnpop	4,496	2.558	0.298	1.305	3.533
House	4,496	0.235	0.501	6.45e − 02	1.289
Innovation	4,496	6.147	13.67	0.0250	166.6
Enterp	4,496	68.36	98.87	1.030	951.7
Ind	4,496	0.724	0.582	0.114	1.168

**Table 3:** Machine learning model parameter setting.

Random forest		XGBoost	
Training time	1.468 s	Training time	1.346 s
Data segmentation	0.7	Data segmentation	0.7
Minimum node splitting	2	Base learner number	100
Minimum leaf node	1	Learning rate	0.1
Maximum depth of tree	10	Sample sign sampling rate	100%
Maximum leaf nodes	50	Tree feature sampling rate	100%
Decision trees number	100	Node feature sampling rate	100%
Put back sampling	True	L2 regular term	1
Out of bag data test	False	Maximum depth of tree	10

The article "Evaluating the Performance of Inclusive Growth Based on the BP Neural Network and Machine Learning Approach" was published in 2022. Journal: Comput Intell Neurosci.

**Table 4:** Machine learning model parameter setting.

CatBoost		LightGBM	
Training time	10.925 s	Training time	0.335 s
Data segmentation	0.7	Data segmentation	0.7
Number of iterations	100	Base learner number	100
Learning rate	0.1	Learning rate	0.1
L2 regular term	1	L2 regular term	1
Maximum depth of tree	10	Sample sign sampling rate	100%
Overfitting test threshold	0	Tree feature sampling rate	100%
Iterations after optimization	20	Maximum depth of tree	10
Data shuffle	NO	Leaf node minimum sample	10

**Table 5:** Machine learning model performance measurement.

Algorithm	Data set	RMSE	MAE	MAPE	*R* ^2^
RF	Training set	0.02	0.03	5.549	0.865
	Testing set	0.034	0.045	8.816	0.266

XGBoost	Training set	0.006	0.003	1.086	0.995
	Testing set	0.006	0.003	1.153	0.989

CatBoost	Training set	0.015	0.011	2.879	0.959
	Testing set	0.014	0.011	3.014	0.895

LightGBM	Training set	0.013	0.01	2.507	0.912
	Testing set	0.013	0.009	2.664	0.917

**Table 6:** Machine learning model performance measurement in different regions.

Region	Data set	RMSE	MAE	MAPE	*R* ^2^
Eastern	Training set	0.001	0	0.115	1
	Testing set	0	0	0.092	1

Central	Training set	0	0.001	0.107	1
	Testing set	0	0	0.093	1

Western	Training set	0.001	0	0.103	1
	Testing set	0	0	0.009	1

**Table 7:** GBDT model performance measurement.

Data set	RMSE	MAE	MAPE	*R* ^2^
Training set	0.014	0.011	2.81	0.972
Testing set	0.013	0.01	2.967	0.937

**Table 8:** Regress results of the econometric model.

	(1)	(2)	(3)	(4)
	IGE	IGE	IGE	IGE
pgdp	0.00000	0.00000^∗∗^	0.00000^∗∗∗^	0.00000^∗^
	(0.00000)	(0.00000)	(0.00000)	(0.00000)
Fd	0.00051	0.00043	0.00049	0.00047
	(0.00052)	(0.00049)	(0.00033)	(0.00046)
Fdi	0.00103	−0.00013	−0.00455^∗∗∗^	0.00095
	(0.00132)	(0.00173)	(0.00100)	(0.00135)
Gove	0.00158	0.00248	0.01339^∗∗^	0.00311
	(0.00354)	(0.00309)	(0.00307)	(0.00324)
Inter	0.02634^∗∗∗^	0.02303^∗∗∗^	0.02072^∗∗∗^	0.02355^∗∗^
	(0.01001)	(0.01528)	(0.00977)	(0.01051)
Lnpop	−0.01748	0.04612	0.03864^∗∗^	0.02098^∗∗^
	(0.02771)	(0.03100)	(0.00339)	(0.00444)
House	−0.00670	−0.00740	−0.02217^∗∗∗^	−0.00831
	(0.00633)	(0.00648)	(0.00511)	(0.00629)
Innovation	0.03302^∗∗∗^	0.03295^∗∗∗^	0.03224^∗∗∗^	0.03295^∗∗∗^
	(0.00044)	(0.00040)	(0.00018)	(0.00029)
Enterp	0.00005	0.00008^∗∗^	0.00009^∗∗∗^	0.00006
	(0.00004)	(0.00004)	(0.00003)	(0.00004)
Ind	0.00052	0.02478^∗∗∗^	0.01229^∗∗∗^	0.00255
	(0.00308)	(0.00293)	(0.00155)	(0.00207)
_cons	0.35371^∗∗∗^	0.16726^∗∗^	0.22540^∗∗∗^	0.25230^∗∗∗^
	(0.06868)	(0.07730)	(0.00874)	(0.01111)
*N*	4496.00000	4496.00000	4496.00000	4496.00000
*R* ^2^	0.70994	0.64938	0.79533	0.75266

Notes: ^∗∗∗^, ^∗∗^, and ^∗^ denote significance at the 1%, 5%, 10% levels, respectively. Robust standard errors in parentheses are clustered by city level.

The article "Evaluating the Performance of Inclusive Growth Based on the BP Neural Network and Machine Learning Approach" was published in 2022. Journal: Comput Intell Neurosci.

## Data Availability

All data included in this study can be obtained from the corresponding author upon request.
